The article "Swarm Intelligence with Adaptive Neuro-Fuzzy Inference System-Based Routing Protocol for Clustered Wireless Sensor Networks" was retracted in 2023. Reasons: signs of a paper mill; suspected computer-generated content; unreliable results or conclusions; concerns about the data.

# Swarm Intelligence with Adaptive Neuro-Fuzzy Inference System-Based Routing Protocol for Clustered Wireless Sensor Networks

**DOI:** 10.1155/2022/7940895

**Published:** 2022-05-13

**Authors:** Feras Mohammed A-Matarneh, Bassam A. Y. Alqaralleh, Fahad Aldhaban, Esam A. AlQaralleh, Anil Kumar, Deepak Gupta, Gyanendra Prasad Joshi

**Affiliations:** ^1^Department of Computer Science, University College of Duba, University of Tabuk, Tabuk 71491, Saudi Arabia; ^2^MIS Department, College of Business Administration, University of Business and Technology, Jeddah 21448, Saudi Arabia; ^3^School of Engineering, Princess Sumaya University for Technology, Amman 11941, Jordan; ^4^Data Science Research Group, School of Computing, DIT University, Dehradun, India; ^5^Department of Computer Science & Engineering, Maharaja Agrasen Institute of Technology, Delhi, India; ^6^Department of Computer Science and Engineering, Sejong University, Seoul 05006, Republic of Korea

## Abstract

Wireless sensor network (WSN) comprises numerous compact-sized sensor nodes which are linked to one another. Lifetime maximization of WSN is considered a challenging problem in the design of WSN since its energy-limited capacity of the inbuilt batteries exists in the sensor nodes. Earlier works have focused on the design of clustering and routing techniques to accomplish energy efficiency and thereby result in an increased lifetime of the network. The multihop route selection process can be treated as an NP-hard problem and can be solved by the use of computational intelligence techniques such as fuzzy logic and swarm intelligence (SI) algorithms. With this motivation, this article aims to focus on the design of swarm intelligence with an adaptive neuro-fuzzy inference system-based routing (SI-ANFISR) protocol for clustered WSN. The proposed SI-ANFISR technique aims to determine the cluster heads (CHs) and optimal routes for multihop communication in the network. To accomplish this, the SI-ANFISR technique primarily employs a weighted clustering algorithm to elect CHs and construct clusters. Besides, the SI-ANFISR technique involves the design of an ANFIS model for the selection process, which make use of three input parameters, namely, residual energy, node degree, and node history. In order to optimally adjust the membership function (MF) of the ANFIS model, the squirrel search algorithm (SSA) is utilized. None of the earlier works have used ANFIS with SSA for the routing process. The design of SSA to tune the MFs of the ANFIS model for optimal routing process in WSN shows the novelty of the study. The experimental validation of the SI-ANFISR technique takes place, and the results are inspected under different aspects. The simulation results highlighted the significant performance of the SI-ANFISR technique compared to the recent techniques with a maximum throughput of 43838 kbps and residual energy of 0.4800J, respectively.

## 1. Introduction

Typically, wireless sensor networks (WSNs) consist of many different entities and are taken into account as the mainstream of sensing in harsh and remote environment locations wherein human interference is impossible. WSN is the self-organizing network domain and thus it comprises several nodes cost-effectively that have the capacity for data processing and wireless communication [1]. WSN is the adaptable lower-cost emerging solution specifically utilized for monitoring the environments [2]. It consists of many smaller devices called sensors with less storage capacity, less computation complexity, and constrained battery power are dispersed in the geographical region for sensing the network state to collect and communicate information [3]. The sensors are distributed in various environments to implement the application, including home automation, industrial, smart grids, habitat monitoring, and military surveillance. Different limitations are enforced on the sensors regarding memory, storage capability, processing power, and energy resources [4].  Figure 1 illustrates the framework of WSN.

The key challenge in WSNs is to expand the lifespan of the network when primary nodes are not able to transfer the information to the sink nodes [5]. In the application of collecting information, all the nodes take responsibility for sensing the data packet to sink nodes. The procedure of gathering information reduces data traffic and stores energy by incorporating several received data packets into individual packets [6]. Therefore, various applications are developed to extend the lifetime of the network. The efficacy of energy is the most important issue in WSNs since sensors are activated by the battery. Consequently, the use of energy can be handled to prolong the lifetime of the system [7]. Clustering is an approach that could alleviate the energy utilization of the sensors by constructing them in an improved method. Considering the constrained battery of sensors, preserving energy is highly significant, or else, the sensors could decrease quickly and that reduces the lifetime and stability period of WSNs [8]. If at all possible, clustering could offer benefits like fault tolerance, scalability, reduced routing delay, data fusion, increased connectivity, stabilized topology, and load balancing.

Several clustering models are introduced and designed in the WSN that depend on the employed model categorized as deterministic and probabilistic systems [9]. The routing methods are significant in WSNs as they offer lesser latency, Quality of Service (QoS), data throughput, and energy consumption. Since WSN is application-specific, several methods are presented to address the problem created when routing data packets. Several computational intelligence (CI) methods including GA, Particle Swarm Optimization (PSO), and neural network (NN), are extensively employed in WSN for several challenges. In general, fuzzy logic (FL) is employed for solving uncertainty in the network. By utilizing FL, a method is enhanced without needing whole data. There are three essential portions comprised of fuzzy decision block (FDB), defuzzifier, and fuzzifier block. FDB is composed of fuzzy inference and rule base system. Fuzzifier blocks convert the crisp input into the suitable fuzzy linguistic parameter. According to the rule base, FDB blocks map the input linguistic variable to the output linguistic variables [10]. At last, defuzzifier blocks convert the fuzzy output into the crisp output through an appropriate defuzzification model.

This study introduces swarm intelligence with an adaptive neuro-fuzzy inference system-based routing (SI-ANFISR) protocol for clustered WSN. The proposed SI-ANFISR technique initially organizes the clusters using the weighted clustering algorithm. Moreover, the SI-ANFISR technique involves the design of the ANFIS model with three input parameters, namely, residual energy (RE), node degree (ND), and node history (NS) to compute the optimal routes to the destination. In order to optimally adjust the membership function (MF) of the ANFIS model, the squirrel search algorithm (SSA) is utilized. The performance analysis of the SI-ANFISR technique takes place and the results are inspected under different aspects.

## 2. Literature Review

Patil and Parveen [11] presented an Adoptive Compressed Sensing (ACS) to resolve problems of hybrid CS. The presented model chooses an ideal size of the cluster and considers the relationship among the several nodes and measurement M. Furthermore, the data collection method uses the traditional Fourier transform to attain better stability with lower computation difficulty. Lastly, an adoptive data recovery approach to clustered WSN is utilized for enhancing the orthogonal matching pursuits.

Kavitha [12] developed a cryptographic-based cluster model to preserve information security through the Optimum Privacy-Multihop Dynamic Clustering Routing Protocol (OP-MDCRP) which enhances energy effectual routing and data privacy for the heterogeneous system that exploits multihop transmission and clustering to decrease the power utilization of sensors and expands the WSN lifetime. According to the region, the source node is combined to create a cluster in the arbitrary system. Also, the method offers higher data security through small key size and Elliptic Curve Integrated Encryption-Key Provisioning Method (ECIES-KPM). Norouzi Shad et al. [13] proposed an Intelligent Decision Support System (IDSS)-based cluster routing method called GA-PSO-SVM, for the IoT perception layer using an SVM-related approach for estimating the location of the node and a hybrid GA-PSO-based method for cluster optimization.

Koyuncu et al. [14] introduced an arithmetical method of Deterministic Energy-Efficient Clustering (DEC)-related multiple tier random possibility protocols for agricultural WSN to improve the lifespan of WSN nodes and comparison of the current DEC method. In the presented method, the election of CH is performed on the basis of the location of the sensors and the energy drain pattern that increases the sensors' lifetime. Rodríguez et al. [15] proposed an energy-effective clustering routing method for WSN-related Yellow Saddle Goatfish Algorithm (YSGA). The method is proposed for intensifying the system lifespan by minimizing power utilization. The networks consider BSs and a collection of CH models. The overall amount of CHs and the optimal selection of CH can be described by the YSGA method, whereas sensors are allocated to its adjacent CH.

Ghaddar et al. [16] presented R-MUCH as a clustering routing method. It is a multiple hop form of the MUCH (Multiple Criteria Cluster Head Delegation-Related Fuzzy Logic) model. CH transmits the information in a multihop manner to the sink by selecting the path which contains the minimum cost in terms of power utilization. R-MUCH is selected for all the CHs. Huamei et al. [17] designed an energy-effective nonuniform cluster routing method for enhancing node energy efficacy and balancing the power utilization in WSN. In addition, a nonuniform cluster network is introduced for reducing the possibility of energy hole existences and improving the CHs selection technique to propose a better-shuffled frog leaping model.

Rodríguez et al. [18] introduced a strong clustering routing method for WSN. The system employs the Locust Search (LS-II) technique for identifying the optimum CHs and determining the amount of CHs. When the CHs are identified, the other sensors are allocated to the adjacent CHs. Brahim et al. [19] suggested that an energy-effective clustering method is very effective when compared to routing methods and provides good coverage of the networks when compared to LEACH. The approach integrates the MCL method for clustering creation, and a novel CHs selection method depends on residual energy and location of sensor nodes.

## 3. System Model

It assumes that the *N* sensor is located randomly from network fields for monitoring the location and their physical feature periodically. All sensors have a neighboring sensor, and it broadcasts information to most neighboring sensors. It can be considered an immobile sensor with equivalent primary energy. The computation ability of all sensors was similar. The symmetric radio connections were regarded amongst some 2 neighboring sensors. The sink was placed inside the network regions. Consider the maximal broadcast of all the sensors is *R*. The adaptive broadcast was regraded by utilizing distance amongst some 2 neighboring sensors. The 1^st^-order radio method for analyzing the energy utilization of presented routing was explained. Assume 7*mm* is the size of the packet from bits. The energy required to broadcast *m* bits of a packet across *d* unit distance amongst a sender sensor and neighboring sensors is written as follows:

(1) $$\begin{array}{c} E_{\text{TX}}\left(m,\;d\right)=\left\{\begin{array}{c} m*E_{\text{elect}}+m*\varepsilon_{\text{fsp}}*d^{2}\text{ if }d<d_{o},\\ m*E_{\text{elect}}+m*\varepsilon_{\text{mpf}}*d^{4}\text{ if }d\geq d_{o}. \end{array}\right. \end{array}$$

For receiving *m* bits of packet, the energy requirement was provided as follows:

(2) $$\begin{array}{c} E_{RX}\left(m\right)=m*E_{\text{Select}},\; \end{array}$$

where *E*_Select_ refers to the statistics on the energy dissipate to transmit electron per bit. Many factors like acceptable bit‐rate, digital coding, and modulation affect the *E*_Select_. The *ε*_fsp_ and *ε*_mpf_ stand for the requirement of energy from the free‐space path and multipath environment, correspondingly. If 2 neighboring sensors whose energy usage has been computed are separated with a distance lesser than or equivalent to $\left(l_{o}=\sqrt{E_{\text{fsp}}/E_{\text{mp}}}\right)$, the radio method executes (1), else (2), for calculating the energy required to transmit the data.

## 4. The Proposed Model

In this study, a new SI-ANFISR technique has been developed for computing the optimal set of multihop routes for intercluster communication in WSN. The proposed SI-ANFISR technique involves three major processes, namely, cluster construction, ANFIS-based route selection, and SSA-based MF selection. The ANFIS model has utilized multiple input parameters for route selection, and the SSA helps to optimally choose the MFs, which results in improved network lifetime.  Figure 2 illustrates the overall working process of the proposed SI-ANFISR technique.

### 4.1. Weighted Clustering Technique

In this study, the SI-ANFISR technique employs a weighted clustering technique involving three input parameters, namely, RE, ND, and NS. In the case of RE, the sensor nodes with maximum energy will be elected as CH. The MF of the RE includes high and low linguistic parameters. The RE defines the ratio of residual energy of node *i* that is related to *E*_*ri*_ and the overall energy of the network *E*_*t*_. It is essential to estimate the RE of all the nodes for every iteration. Consequently, a balanced energy depletion can be accomplished in the network.

(3) $$\begin{array}{c} \text{Residual energy}=\overset{n}{\underset{i=1}{\sum }}\frac{E_{ri}}{E_{t}}. \end{array}$$

Next, the NSs are related to the iterations. The CHs are chosen with maximum iterations; in new iterations, the CHs are chosen with the low ability of the node.

(4) $$\begin{array}{c} \text{Node histories }=\;1-\lambda H^{t-1}\left(n\right)-\lambda^{2}H^{t-2}\left(n\right),\ldots ,\;\lambda^{r}H^{t-r}\left(n\right)\;, \end{array}$$

where *t* indicates the present round and the earlier round is represented as *t *−* *1, and in *r* preceding rounds, *t *−* r* identifies the round number. *λ* can be defined using the coefficient values of the history nodes, and the element *H*^*t*−*r*^ is either 0 or 1. Finally, the ND of a chosen CH is as follows:

(5) $$\begin{array}{c} ND=\frac{T}{N}, \end{array}$$

where the number of neighboring nodes is elected as CH, which can be defined by T. For every node, a weight value *P*_*i*_ is

(6) $$\begin{array}{c} P_{i}=w_{1}*RE_{i}+w_{2}*ND_{i}+w_{3}*NS_{i}, \end{array}$$

where *w*_1_, *w*_2_, and *w*_3_ denote the coefficient values. Hence,

(7) $$\begin{array}{c} w_{1}+w_{2}+w_{3}=1. \end{array}$$

### 4.2. Design of the ANFIS Model for the Routing Process

Once the clusters are constructed, the next stage is to derive optimal routes for intercluster communication using the ANFIS model. It receives the input parameters as RE, ND, and NS to compute optimal paths. The ANFIS is established by Jangthat mentions the combination of FL and ANN for creating the important processing equipment [20]. Indeed, 2 rules are generated to all inputs with a maximal value equivalent to 1 and minimal value equivalent to 0. It is a multilayer feed‐forward network (MLFN) in that all nodes obtain the particular function on the input signal.

The square and circle node symbols are employed for characterizing distinct learning parameters. The parameter is altered for achieving the chosen input and output attributes based on the learning rule. The parameters energy, resource utilization, computation cost, makespan, and memory are utilized as input for the ANFIS technique. The resultant parameter is tuned by utilizing the BWO technique for obtaining better outcomes. The BWO technique employed during this artifact for supporting ANFIS adjusts the parameter of membership functions (MF). The fuzzy inference system has been considered that has 5 layers of adaptive network with 2 inputs *a* and *b* and only one output *c*. The node in *j*^*th*^ place of *l*^*th*^ layer has been demonstrated as *O*_*l*,*j*_, and the function of the node from the same layer of an identical function family is demonstrated as follows.

Layer 1: Layer 1 signifies the input layer, and all nodes *j* from Layer 1 imply the square node by node functions. *O*_*l*,*j*_ stands for the MF of *X*_*j*_ and defines the obtainable degree that persuades the quantifier *X*_*j*_. Usually, the bell‐shaped MF was selected as input of MF by maximal equivalent to 1 and the minimal equivalent to 0.

(8) $$\begin{array}{c} O_{1,\text{j}}=\mu X_{j}\left(a\right)\text{for }j=1,2,\\ \mu X_{j}\left(a\right)=\frac{1}{1+{\left[{\left(a-z_{j}/x_{j}\right)}^{2}\right]}^{y_{j}}}, \end{array}$$

where *x*_*j*_, *y*_*j*_, and *z*_*j*_ signifies the parameters, *y* stands for the positive value, and *z* implies the curve center.

Layer 2: all the nodes under this layer signify the square node, obvious as Π that generates the incoming signal and forwards the outcome product [21].

(9) $$\begin{array}{c} O_{2,j}=w_{j}=\mu X_{j}\left(a\right)\times \mu Y_{j}\left(b\right)\text{for }j=1,2. \end{array}$$

Layer 3: all the nodes under this layer represent square nodes, noticeable as M. The *j*^*th*^ node estimates the ratio of *j*^*th*^ rule firing strength to further of every rule to fire strength based on the formula. The outcome of this layer can be named as normalization firing strength.

(10) $$\begin{array}{c} O_{3,j}=\bar{w}=\frac{w_{j}}{w_{1}+w_{2}}\text{ for }j=1,2\;. \end{array}$$

Layer 4: all the nodes *j* under this layer signify the square node by node function. The attribute under this layer is demonstrated as the following attribute:

(11) $$\begin{array}{c} O_{4,j}={\bar{w}}_{j}f_{j}={\bar{w}}_{j}\left(p_{j}+q_{j}+r_{j}\right), \end{array}$$

where *p*_*j*_, *q*_*j*_, and *r*_*j*_ stand for the attribute.

Layer 5: the single node from Layer 5 signifies the circle node, obvious as Σ that estimates the entire outcome in addition to every the incoming signal according to the following formula:

(12) $$\begin{array}{c} O_{5,j}=\underset{j}{\sum }{\bar{w}}_{j}f_{j}=\frac{\sum_{j=1}w_{j}f}{\sum_{j=1}w_{j}}=\text{ output}. \end{array}$$

### 4.3. SSA-Based Parameter Optimization

In order to optimally tune the MF of the ANFIS model, the SSA is used which thereby improves the overall performance of the ANFIS model. Initially, the SSA tries to randomly generate a population initialization that represents the location of the squirrel [22]. In the SSA, the position of all the squirrels is described by a *d* dimension vector. This process considers the position of *n* squirrels in a 2D matrix as follows:

(13) $$\begin{array}{c} FS=\begin{array}{ccccc} S11 & S12 & \cdots & \cdots & S1d\\ S21 & S22 & \cdots & \cdots & S2d\\ \cdots & \cdots & \cdots & \cdots & \cdots \\ \cdots & \cdots & \cdots & \cdots & \cdots \\ Sn1 & Sn2 & \cdots & \cdots & \text{Snd} \end{array}\;.\; \end{array}$$

Here, *S*_*i*_ is the *i*^*th*^ flying squirrel, and *S*_*ij*_ is its *j*^*th*^ dimension.

(14) $$\begin{array}{c} S_{ij}=S_{l}+\text{Rand}\left(0,1\right)*\left(S_{u}-S_{l}\right). \end{array}$$

Here, *S*_*u*_ and *S*_*l*_ are upper and lower limits of *S*_*i*_ in *j*^*th*^ parameter and Rand (0, 1) denotes a function to generate arbitrary values within [0,1]. As well, the fitness of position for every *S*_*i*_ is computed by the following matrix:

(15) $$\begin{array}{c} \text{Fit}=\left\{\begin{array}{ccc} F\left(S11\right. & S12 & S1d\\ F\left(S21\right. & S22 & S2d\\ \cdots & \cdots & \cdots \\ F\left(Sn1,\cdots \right) & Sn2 & \cdots \text{Snd} \end{array}\right\},\\ \left\{\begin{array}{c} F\left(S11,\;S12,\ldots ,S1d\right.\;\\ F\left(S21,\;S22,\ldots ,S2d\right.\\ \cdots \\ \;\cdots \\ F\left(Sn1,Sn2,\ldots ,Snd\right. \end{array}\right\}. \end{array}$$

Here, *F* shows the fitness function. After calculating the fitness value of every *S*_*i*_, they are arranged in ascending order. The SSA categorizes the squirrel into three major classes. As well, to fulfill the energy requirement, some squirrels randomly move toward the hickory nut tree and others move towards the acorn nut tree, based on the existence of distinct predators. The flying squirrel is on acorn nut tree and moves toward the hickory tree which can be computed by the following equation:

(16) $$\begin{array}{c} S_{at}^{t+1}=\left\{\begin{array}{cc} S_{at}^{t}+dg*Gc*\left(S_{ht}^{t}-S_{at}^{t}\right) & R_{1}\geq P_{dp}\\ \text{random} & \text{otherwise} \end{array}\right\}. \end{array}$$

Here, *t* represents the existing iteration, *dg* denotes random gliding distance, *P*_*dp*_ indicates predator existence probability, *R*_1_ indicates an arbitrary value within [0, 1], and *S*_*ht*_ shows the position of flying squirrels that reached the hickory tree. The balance between exploitation and exploration can be attained by the gliding constant *G*_*c*_ in the arithmetical model is formulated in the following equation [23]:

(17) $$\begin{array}{c} S_{at}^{t+1}=\left\{\begin{array}{cc} S_{nt}^{t}+dg*Gc*\left(S_{at}^{t}-S_{nt}^{t}\right) & R_{2}\geq P_{dp}\\ \text{random} & \text{otherwise} \end{array}\right\}\;. \end{array}$$

Now, *R*_2_ represents an arbitrary value in [0, 1]. As well, few squirrels on the normal tree might move to hickory nut trees for storing hickory nuts. This can be expressed by the following equation:

(18) $$\begin{array}{c} S_{at}^{t+1}=\left\{\begin{array}{cc} S_{at}^{t}+dg*Gc*\left(S_{ht}^{t}-S_{at}^{t}\right)\; & R_{3}\geq Pd\\ \text{random} & \text{otherwise} \end{array}\right\}. \end{array}$$

Let *R*_3_ be an arbitrary value within [0, 1] as well as the predator probability *P*_*dp*_ is assumed as 0.1.  Algorithm 1 shows the pseudocode of SSA.

## 5. Experimental Validation

The performance validation of the SI-ANFISR technique is simulated using the MATLAB tool. The results are examined under two scenarios: 200 nodes and 500 nodes. The node deployment of two scenarios is shown in Figure 3 with BS at the center. A comparative analysis is made with existing methods such as exponentially-ant lion whale optimization algorithm (E-ALWO) [24], Energy-Efficient Scalable Routing Algorithm (EESRA) [25], multidimensional scaling map (MDS-MAP) [26], grey wolf optimization, and Routing Protocol for low power and Lossy networks (RPL) [27].

Table 1 and Figure 4 offer a comparative study of the SI-ANFISR technique with other techniques under 200 nodes. On examining the results in terms of delay, it is apparent that the SI-ANFISR technique has gained minimal delay under all rounds. For instance, with 200 rounds, the SI-ANFISR technique has offered the least delay of 0.1633 s whereas the E-ALWO, RPL, MDS-MAP, EESRA, and GWO techniques have obtained an increased delay of 0.1727 s, 0.2073 s, 0.2240 s, 0.2276 s, and 0.2356 s, respectively. Similarly, with 1000 rounds, the SI-ANFISR technique has provided decreased delay of 0.1862 s, whereas the E-ALWO, RPL, MDS-MAP, EESRA, and GWO techniques have attained an increased delay of 0.2135 s, 0.2549 s, 0.2662 s, 0.2702 s, and 0.2774 s, respectively.

On inspecting the performance with respect to RE, the results notified the betterment of the SI-ANFISR technique with increased RE. For instance, with 200 rounds, the SI-ANFISR technique has reached a higher RE of 0.4421J, whereas the E-ALWO, RPL, MDS-MAP, EESRA, and GWO techniques have attained a lower RE of 0.4138J, 0.2462J, 0.3699J, 0.3699J, and 0.3674J, respectively. Similarly, with 1000 rounds, the SI-ANFISR system has attained a superior RE of 0.1985J, whereas the E-ALWO, RPL, MDS-MAP, EESRA, and GWO algorithms have obtained a minimum RE of 0.1122J, 0.0003J, 0.0825J, 0.0013J, and 0.0026J, correspondingly.

On examining the performance with respect to throughput, the results notified the betterment of the SI-ANFISR technique with higher RE. For instance, with 200 rounds, the SI-ANFISR method has gained a superior throughput of 10124 kbps whereas the E-ALWO, RPL, MDS-MAP, EESRA, and GWO techniques have attained a lower throughput of 8120 kbps, 5881 kbps, 7295 kbps, 5998 kbps, and 4938 kbps, correspondingly. Likewise, with 1000 rounds, the SI-ANFISR algorithm has reached higher throughput of 43838 kbps, whereas the E-ALWO, RPL, MDS-MAP, EESRA, and GWO systems have gained a minimum throughput of 42895 kbps, 34054 kbps, 32757 kbps, 33700 kbps, and 30164 kbps, correspondingly.

Table 2 and Figure 5 provide a comparative study of the SI-ANFISR algorithm with other methods under 500 nodes. On investigating the outcomes with respect to delay, it can be clear that the SI-ANFISR technique has gained minimal delay under all rounds. For instance, with 200 rounds, the SI-ANFISR algorithm has an obtainable worse delay of 0.1843 s, whereas the E-ALWO, RPL, MDS-MAP, EESRA, and GWO techniques have obtained an increased delay of 0.1997 s, 0.2304 s, 0.2486 s, 0.2595 s, and 0.2711 s, correspondingly. At the same time, with 1000 rounds, the SI-ANFISR technique has provided decreased delay of 0.2075 s whereas the E-ALWO, RPL, MDS-MAP, EESRA, and GWO methods have reached a maximum delay of 0.2396 s, 0.2854 s, 0.2854 s, 0.2865 s, and 0.3053 s, correspondingly.

On analyzing the performance with respect to RE, the results notified the betterment of the SI-ANFISR technique with increased RE. For instance, with 200 rounds, the SI-ANFISR algorithm has reached a maximum RE of 0.4800J whereas the E-ALWO, RPL, MDS-MAP, EESRA, and GWO techniques have attained minimal RE of 0.4540J, 0.2895J, 0.4149J, 0.4127J, and 0.4070J, correspondingly. Afterward, with 1000 rounds, the SI-ANFISR system has reached a maximum RE of 0.2340J, whereas the E-ALWO, RPL, MDS-MAP, EESRA, and GWO techniques have attained reduced RE of 0.1471J, 0.0340J, 0.1152J, 0.0409J, and 0.0368J, correspondingly.

Moreover, on examining the performance with respect to throughput, the results notified the betterment of the SI-ANFISR algorithm with increased RE. For instance, with 200 rounds, the SI-ANFISR technique has reached a superior throughput of 10124 kbps, whereas the E-ALWO, RPL, MDS-MAP, EESRA, and GWO techniques have achieved a lower throughput of 8120 kbps, 5881 kbps, 7295 kbps, 5998 kbps, and 4938 kbps, respectively. Followed by, with 1000 rounds, the SI-ANFISR technique has reached a higher throughput of 43838 kbps, whereas the E-ALWO, RPL, MDS-MAP, EESRA, and GWO techniques have attained a decreased throughput of 42895 kbps, 34054 kbps, 32757 kbps, 33700 kbps, and 30164 kbps, correspondingly.

Next, the TPR analysis of the SI-ANFISR technique with existing techniques is made in Table 3 and Figure 6. The results reported the betterment of the SI-ANFISR technique under all nodes. For instance, with 200 nodes, the SI-ANFISR technique has resulted in a higher TPR of 155512 bytes, whereas the E-ALWO, RPL, MDS-MAP, EESRA, and GWO techniques have attained a lower TPR of 131445, 103476, 64147, 34286, and 9328 bytes, respectively. In addition, with 500 nodes, the SI-ANFISR method has resulted in a higher TPR of 172002 bytes, whereas the E-ALWO, RPL, MDS-MAP, EESRA, and GWO methodologies have attained a reduced TPR of 151501, 117629, 86431, 57462, and 19133 bytes, correspondingly.

Finally, a brief routing overhead (ROH) analysis of the SI-ANFISR technique with recent approaches is shown in Table 4 and Figure 7 [24]. The results exhibited the improvement of the SI-ANFISR technique over the recent methods with a minimum amount of ROH under varying node counts. For instance, with 200 nodes, the SI-ANFISR technique has offered a lower ROH of 12%, whereas the E-ALWO, RPL, MDS-MAP, EESRA, and GWO techniques have provided a higher ROH of 20%, 36%, 45%, 58%, and 68%, respectively.

Similarly, with 500 nodes, the SI-ANFISR technique has accomplished a minimal ROH of 16%, whereas the E-ALWO, RPL, MDS-MAP, EESRA, and GWO techniques have resulted in a maximum ROCH of 25%, 38%, 54%, 63%, and 72%, respectively. After examining the results and discussion, it is verified that the SI-ANFISR technique has resulted in effective performance over the recent approaches.

## 6. Conclusion

In this study, a new SI-ANFISR technique has been developed for computing the optimal set of multihop routes for intercluster communication in WSN. The proposed SI-ANFISR technique involves three major processes, namely, cluster construction, ANFIS-based route selection, and SSA-based MF selection. The ANFIS model has utilized multiple input parameters for route selection, and the SSA helps to optimally choose the MFs, which results in improved network lifetime. The performance analysis of the SI-ANFISR technique takes place, and the results are inspected under different aspects. The simulation results highlighted the significant performance of the SI-ANFISR technique compared to the recent technique's maximum throughput of 43838 kbps and RE of 0.4800J, respectively. Therefore, the SI-ANFISR technique can be treated as an effective solution to increase the lifetime of the WSN. In the future, data compression approaches can be integrated into the clustering model to boost energy efficacy in WSN.

## Figures and Tables

**Figure 1:** WSN structure.

**Figure 2:** Working process of the SI-ANFISR technique.

**Figure 3:** Node deployment: (a) 200 nodes; (b) 500 nodes.

**Figure 4:** Result analysis of the SI-ANFISR technique under 200 nodes.

**Figure 5:** Result analysis of the SI-ANFISR technique under 500 nodes.

**Figure 6:** TPR analysis of the SI-ANFISR technique with existing methods.

**Figure 7:** ROH analysis of the SI-ANFISR technique with existing methods.

**Algorithm 1:** Pseudocode of SSA.

**Table 1:** Result analysis of the SI-ANFISR technique with existing methods under 200 nodes.

No. of rounds	SI-ANFISR	E-ALWO	RPL	MDS-MAP	EESRA	GWO
Delay (sec)						
200	0.1633	0.1727	0.2073	0.2240	0.2276	0.2356
400	0.1684	0.1785	0.2142	0.2291	0.2342	0.2400
600	0.1716	0.1840	0.2193	0.2342	0.2382	0.2440
800	0.1815	0.1887	0.2265	0.2404	0.2458	0.2553
1000	0.1862	0.2135	0.2549	0.2662	0.2702	0.2774

Residual energy (J)						
200	0.4421	0.4138	0.2462	0.3699	0.3699	0.3674
400	0.3828	0.3313	0.1547	0.2668	0.2410	0.2372
600	0.3042	0.2578	0.1006	0.2101	0.1186	0.1173
800	0.2230	0.1792	0.0477	0.1354	0.0026	0.0245
1000	0.1985	0.1122	0.0003	0.0825	0.0013	0.0026

Throughput (kbps)						
200	10124	8120	5881	7295	5998	4938
400	18022	16018	11892	14722	11892	9771
600	28396	23798	17315	20616	16843	15075
800	37826	32757	33700	26745	33229	26863
1000	43838	42895	34054	32757	33700	30164

**Table 2:** Result analysis of the SI-ANFISR technique with existing methods under 500 nodes.

No. of rounds	SI-ANFISR	E-ALWO	RPL	MDS-MAP	EESRA	GWO
Delay (sec)						
200	0.1843	0.1997	0.2304	0.2486	0.2595	0.2711
400	0.1918	0.2064	0.2449	0.2571	0.2543	0.2739
600	0.1990	0.2202	0.2466	0.2597	0.2726	0.2808
800	0.2090	0.2134	0.2554	0.2665	0.2761	0.2941
1000	0.2075	0.2396	0.2854	0.2865	0.3053	0.3122

Residual energy (J)						
200	0.4800	0.4540	0.2895	0.4149	0.4127	0.4070
400	0.4237	0.3617	0.1977	0.3088	0.2753	0.2702
600	0.3408	0.2970	0.1325	0.2425	0.1489	0.1503
800	0.2625	0.2258	0.0777	0.1765	0.0457	0.0596
1000	0.2340	0.1471	0.0340	0.1152	0.0409	0.0368

Throughput (kbps)						
200	10124	8120	5881	7295	5998	4938
400	18022	16018	11892	14722	11892	9771
600	28396	23798	17315	20616	16843	15075
800	37826	32757	33700	26745	33229	26863
1000	43838	42895	34054	32757	33700	30164

**Table 3:** Analysis on total packets received of the SI-ANFISR technique with existing methods.

Total packets received by BS (byte)		
Methods	200 nodes	500 nodes
SI-ANFISR	155512	172002
E-ALWO	131445	151501
RPL	102476	117629
MDS-MAP	64147	86431
EESRA	34286	57462
GWO	9328	19133

**Table 4:** Routing overhead analysis of the SI-ANFISR technique with existing approaches.

Routing overhead (%)		
Methods	200 nodes	500 nodes
SI-ANFISR	12	16
E-ALWO	20	25
RPL	36	38
MDS-MAP	45	54
EESRA	58	63
GWO	68	72

## Data Availability

No data were used to support this study.

## References

[1] Raja Basha A. (2022). A review on wireless sensor networks: routing. *Wireless Personal Communications*.

[2] Ramteke R., Singh S., Malik A. (2022). Optimized routing technique for IoT enabled software-defined heterogeneous WSNs using genetic mutation based PSO. *Computer Standards & Interfaces*.

[3] Chang L., Li F., Niu X., Zhu J. (2022). On an improved clustering algorithm based on node density for WSN routing protocol. *Cluster Computing*.

[4] Mohemed R. E., Saleh A. I., Abdelrazzak M., Samra A. S. (2017). Energy-efficient routing protocols for solving energy hole problem in wireless sensor networks. *Computer Networks*.

[5] Arjunan S., Pothula S., Ponnurangam D. (2018). F5N-based unequal clustering protocol (F5NUCP) for wireless sensor networks. *International Journal of Communication Systems*.

[6] Arjunan S., Pothula S. (2019). A survey on unequal clustering protocols in wireless sensor networks. *Journal of King Saud University - Computer and Information Sciences*.

[7] Famila S., Jawahar A., Sariga A., Shankar K. (2020). Improved artificial bee colony optimization based clustering algorithm for SMART sensor environments. *Peer-to-Peer Networking and Applications*.

[8] Ismail A. S., Wang X., Hawbani A., Alsamhi S., Abdel Aziz S. (2022). Routing protocols classification for underwater wireless sensor networks based on localization and mobility. *Wireless Networks*.

[9] Venkataraman R. (2019). EODC: an energy optimized dynamic clustering protocol for wireless sensor network using PSO approach. *International Journal of Computers, Communications & Control*.

[10] Ruan D., Huang J. (2019). A PSO-based uneven dynamic clustering multi-hop routing protocol for wireless sensor networks. *Sensors*.

[11] Patil N. S., Parveen A. (2021). ACS LEACH protocol using optimized clustering and improved orthogonal matching pursuit in WSN. *International Journal of Information Technology*.

[12] Kavitha V. (2021). Privacy preserving using multi-hop dynamic clustering routing protocol and elliptic curve cryptosystem for WSN in IoT environment. *Peer-to-Peer Networking and Applications*.

[13] Norouzi Shad M., Maadani M., Nesari Moghadam M. (2021). GAPSO-SVM: an IDSS-based energy-aware clustering routing algorithm for IoT perception layer. *Wireless Personal Communications*.

[14] Koyuncu H., Tomar G. S., Sharma D. (2020). A new energy efficient multitier deterministic energy-efficient clustering routing protocol for wireless sensor networks. *Symmetry*.

[15] Rodríguez A., Del-Valle-Soto C., Velázquez R. (2020). Energy-efficient clustering routing protocol for wireless sensor networks based on yellow saddle goatfish algorithm. *Mathematics*.

[16] Ghaddar A., Ghosn M. H., Mitton N. (2020). R-MUCH: a clustering routing algorithm using fuzzy logic for WSNs. *IOP Conference Series: Materials Science and Engineering*.

[17] Huamei Q., Chubin L., Yijiahe G., Wangping X., Ying J. (2021). An energy‐efficient non‐uniform clustering routing protocol based on improved shuffled frog leaping algorithm for wireless sensor networks. *IET Communications*.

[18] Rodríguez A., Pérez-Cisneros M., Rosas-Caro J. C., Del-Valle-Soto C., Gálvez J., Cuevas E. (2021). Robust clustering routing method for wireless sensor networks considering the Locust search scheme. *Energies*.

[19] Brahim M. T., Abbad H., Boukil-Hacene S. (2021). A low energy mcl-based clustering routing protocol for wireless sensor networks. *International Journal of Wireless Networks and Broadband Technologies*.

[20] Yi J.-H., Deb S., Dong J., Alavi A. H., Wang G.-G. (2018). An improved NSGA-III algorithm with adaptive mutation operator for Big Data optimization problems. *Future Generation Computer Systems*.

[21] Nanjappan M., Natesan G., Krishnadoss P. (2021). An adaptive neuro-fuzzy inference system and black widow optimization approach for optimal resource utilization and task scheduling in a cloud environment. *Wireless Personal Communications*.

[22] Jain M., Singh V., Rani A. (2019). A novel nature-inspired algorithm for optimization: squirrel search algorithm. *Swarm and Evolutionary Computation*.

[23] Zheng T., Luo W. (2019). An improved squirrel search algorithm for optimization. *Complexity*.

[24] SureshKumar K., Vimala P. (2021). Energy efficient routing protocol using exponentially-ant lion whale optimization algorithm in wireless sensor networks. *Computer Networks*.

[25] Ahmed Elsmany E. F., Omar M. A., Wan T.-C., Altahir A. A. (2019). EESRA: energy efficient scalable routing algorithm for wireless sensor networks. *IEEE Access*.

[26] Beheshtiasl A., Ghaffari A. (2019). Secure and trust-aware routing scheme in wireless sensor networks. *Wireless Personal Communications*.

[27] Heurtefeux K., Menouar H. Experimental evaluation of a routing protocol for wireless sensor networks: RPL under study.

